The article "Comparison of Affected-Vertebra Fixation of Cortical Bone Trajectory Screw and Pedicle Screw for Lumbar Tuberculosis: A Minimum 3-Year Follow-Up" was published in 2022. Journal: Biomed Res Int.

# Comparison of Affected-Vertebra Fixation of Cortical Bone Trajectory Screw and Pedicle Screw for Lumbar Tuberculosis: A Minimum 3-Year Follow-Up

**DOI:** 10.1155/2022/6312994

**Published:** 2022-07-21

**Authors:** Peng Zhang, Jiekai Ye, Lixia Huang, Xiaozhang Ying, Bo Zhu, Yanghui Jin, Jun Fei, Shiyuan Shi, Qi Zheng

**Affiliations:** Affiliated Hangzhou Chest Hospital, Zhejiang University School of Medicine, Hangzhou, China

## Abstract

**Purpose:**

This study is aimed at comparing the clinical efficacy of cortical bone trajectory (CBT) screw fixation and pedicle screw (PS) fixation of the affected vertebrae in lumbar tuberculosis.

**Methods:**

We retrospectively analyzed the outcomes in 52 patients (27 cases in the CBT group, 25 cases in the PS group) with lumbar TB who underwent posterior affected-vertebra fixation combined with anterior debridement and bone grafting. The intraoperative blood loss, operative time, visual analog scale (VAS) scores for incision pain and leg pain, Japanese Orthopedic Association (JOA) score, bone grafting fusion, and complications were recorded.

**Results:**

All patients were followed up for 35-52 months and achieved good clinical outcomes. There were no differences between the two groups in the operative time, intraoperative blood loss, JOA score, bone grafting fusion, and complications. However, there was a significant difference between the two groups in VAS scores for incision pain on the 1st day and 3rd day after surgery. At the last follow-up, JOA scores were significantly improved in both groups compared to the preoperation.

**Conclusion:**

This retrospective study confirmed that both the affected-vertebra CBT screw fixation and PS fixation for lumbar TB via posterior and anterior approaches could achieve satisfactory outcomes, while the former resulted in better improvement for postoperative VAS scores.

## 1. Introduction

Spinal tuberculosis (TB) is a common form of extrapulmonary tuberculosis, with the highest incidence of lumbar TB [1]. Spinal TB severely damages the adjacent vertebral bodies and intervertebral disc space, resulting in neurological deficits, kyphotic deformities, and paraplegia [2]. The current treatment of spinal TB includes antituberculosis drugs and surgical intervention. When there is vertebral instability, chemotherapy failure, progressive deformity, neurological injury, or large abscess, surgery for spinal TB is required. Various surgical approaches have been widely used to treat spinal TB, including the anterior and posterior approaches [3]. Since spinal TB mainly leads to the destruction of anterior vertebral columns and the formation of presacral or iliopsoas abscess, many surgeons favor the posterior fixation combined with anterior debridement and bone grafting [4, 5], which provides a direct and optimal view to facilitating thorough debridement.

Using a screw fixation system is a crucial way to reconstruct spinal TB stability, including long-segment fixation and short-segment fixation [6, 7]. Both the two fixation methods can effectively restore spinal TB stability; however, these methods not only impair the normal unit motor function but also accelerate the degradation of adjacent segments [8]. Realizing these problems, Shi et al. [9] proposed pedicle screw (PS) fixation of the affected vertebrae (termed affected-vertebra fixation) that maximally maintains the spinal motor function and achieves good outcomes.

The PS fixation method has been accepted as the gold standard technique due to its excellent biomechanical strength in reconstructing the stability of the spine [10]. The traditional insertion pathway for PS follows a lateral path along the axial plane, which causes the contact strength of the screw-bone interface to mainly depend on the quality of cancellous bone [11]. Therefore, patients with osteoporosis are at risk of loosening with the pedicle screws [12]. Undoubtedly, this situation is also likely to occur in TB patients with the damaged anterior-middle vertebral columns. The cortical bone trajectory (CBT) screw fixation diminishes this complication because both the entry trajectories of the CBT screw in the sagittal and axial plane significantly engage cortical bone and increase the contact strength of the screw-bone interface [13].

We retrospectively analyzed the outcomes in patients with lumbar TB who underwent posterior affected-vertebra fixation combined with anterior debridement and bone grafting. Thus, this study is aimed at comparing the clinical efficacy of CBT screw fixation and PS fixation for lumbar tuberculosis.

## 2. Materials and Methods

### 2.1. Clinical Data

We retrospectively analyzed the outcomes in 52 patients (27 cases in the CBT group, 25 cases in the PS group) with lumbar TB who underwent posterior affected-vertebra fixation combined with anterior debridement and bone grafting from January 2017 to May 2019. Demographic and clinical characteristics like sex, age, and the number of affected vertebras were collected at baseline (Table 1). This study was approved by the Ethics Committee of Affiliated Hangzhou Chest Hospital, Zhejiang University School of Medicine (Hangzhou, China). The written informed consent was obtained from each patient.

The diagnosis of lumbar TB was based on the medical history, clinical symptoms, radiographic examination, and laboratory examination. Patients were included in the study if they had suggestive symptoms of spinal TB like low back pain and restricted lumbar vertebral function and general symptoms with fatigue, night sweats, low fever, and weight loss. Radiological alterations that were considered as suggestive of spinal TB were osteoclasia and sequestra and psoas abscesses or abscesses near the affected vertebrae. According to the previous study [14], the following diagnostic methods were used to confirm TB in this study, including acid-fast staining and microbiological examination of the focal tissue, rapid liquid culture using the BACTEC MGIT 960 system (BD Biosciences, USA), and GeneXpert assay (MTB/RIF, BD, USA).

Patients with spinal instability, spinal nerve dysfunction, and severe back pain were selected. Patients with severe kyphosis deformity (>60°), destruction of the pedicle of a vertebra, surgical contraindications, and mental illness were excluded. Preoperatively, all patients received at least 2 weeks of antituberculosis chemotherapy with rifampicin (0.45 g/kg/d), ethambutol (0.75 g/kg/d), isoniazid (0.3 g/kg/d), and pyrazinamide (1.5 g/kg/d) [15]. During medication, we used glycyrrhizic acid as a liver protection drug, which has been clinically proven to be effective on preventing antituberculosis drug-induced liver injury [16]. After the patient's general condition had improved, a feasible surgical plan for each patient was carried out.

### 2.2. Surgical Procedure

After general anesthesia, the routine posterior midline approach was conducted to expose the affected segments. In the two groups, the appropriate PS and CBT screws were placed into the pedicle of the affected vertebrae. After that, the appropriate length of titanium rod was selected and fixed with screws. After internal fixation, the patients were turned to a semilateral position, and a retroperitoneal approach through a small abdominal incision in the midaxillary line was made. Then, the anterior debridement and bone grafting were performed after the exposure of the affected vertebrae.

### 2.3. Radiological and Clinical Evaluations

All patients were postoperatively rested in bed for two weeks and received antituberculosis and liver protection drugs, after which they could gradually walk under a protective load. Each patient visited our hospital monthly in the first six postoperative months postdischarge and then once a year. Blood indicators, including liver function, erythrocyte sedimentation rate (ESR), and C-reactive protein level (CRP), were monitored carefully every month. X-rays, CT reconstruction, and MRI were obtained at each follow-up visit. After surgery, we usually keep patients on antituberculosis chemotherapy for 12 months to consolidate the treatment effect [2]. Finally, the decision of antituberculosis drug withdrawal requires a combination of patient complaints and blood indicators (liver function, ESR, and CRP) and imaging examination [1, 2]. When the patient has no local pain or tenderness and no cold abscess or sinus formation, blood indicators returned to normal, and imaging examination confirmed that the lesion was healing, and there is complete bone graft fusion, a decision can be made to stop the antituberculosis drug. The various indicators of intraoperative blood loss, operative time, visual analog scale (VAS) score for incision pain and leg pain, Japanese Orthopedic Association (JOA) score, bone grafting fusion, and complications were observed and compared.

### 2.4. Statistical Analysis

Statistical data analyses were performed using SPSS 16.0 (IBM, USA). All measurement data were expressed as mean ± standard deviation. Fisher's exact probability test and independent-samples *t*-test and logistic regression analysis were performed in the present research using SPSS software. *p* < 0.05 was considered significant.

## 3. Results

All 52 patients had complete epidemiological and clinical data and total radiographic measurements available for analysis. There were no significant differences in the sex, age, or the number of affected vertebrae of the patients (Table 1). The majority of identified TB cases in our study were confirmed by acid-fast staining and microbiological examination of the focal tissue, rapid liquid culture using the BACTEC MGIT 960 system (BD Biosciences, USA), and GeneXpert assay (MTB/RIF, BD, USA), accounting for more than 90% of the identified TB cases.

All patients were followed up for 35-52 months. Average operative time and intraoperative blood loss are shown in Table 2. VAS scores for incision and leg pain postoperation are shown in Figure 1. During the follow-up period, no loosening of CBT screw fixation occurred, while one case of PS screw fixation was loosened and the bone graft fused completely after revision surgery. All patients in the CBT and PS groups had good bone grafting fusion, with an average fusion time of 3.9 and 4.3 months, respectively (Table 2). At the last follow-up, JOA scores were significantly improved in both groups compared to the preoperation (Table 3). The mean duration of TB treatment in this study was 12.6 months.

All patients have no intraoperative complications, such as nerve and enormous blood vessel damage. One case of aseptic fat liquefaction occurred in the CBT group after surgery, cured by thorough debridement and drainage. One case of iliac abscess occurred in the PS group after surgery, which was cured by needle aspiration under B-mode ultrasound guidance and catheter flushing and drainage. The typical cases are shown in Figures 2 and 3.

## 4. Discussion

In spinal TB, the incidence of lumbar TB is the highest, while spine surgery combined with antituberculosis chemotherapy can achieve satisfactory results [17, 18]. Spine surgical intervention is an effective method to rebuild spine's stability and relieve nerve compression, effectively controlling the disease and shortening the treatment cycle. When vertebral bone destruction involves anterior and middle columns simultaneously, the presacral or iliopsoas abscess, neurological injury, and vertebral instability make it very difficult to debride completely and effectively fix via a single approach [19, 20]. Therefore, posterior screw fixation combined with complete anterior debridement and bone grafting to treat lumbar TB can compensate for the disadvantages of a single approach.

At present, both long- and short-segment fixations are widely used to reconstruct the stability of spinal TB [21, 22]. Although these methods provide strong fixation, the motor function of the normal unit is sacrificed, which accelerates the degradation of adjacent segments. Clinical and biomechanical assessments have shown that the more the fixed vertebrae, the greater the possibility of degeneration of the adjacent vertebrae [23, 24]. However, the debridement and fixation of the only affected vertebrae, which do not involve adjacent normal vertebrae, maximally maintain the normal motor function, reduce adjacent vertebral degeneration, and achieve good outcomes [1].

Posterior PS fixation has been commonly used in spinal surgery due to its excellent biomechanical strength to reconstruct the stability of the spine [25, 26]. It is reported that posterior PS fixation of the affected vertebrae of spinal TB maximally maintains the spinal motor function and achieves good outcomes [9]. The traditional insertion pathway for PS follows a lateral path along the axial plane, which causes the contact strength of the screw-bone interface mainly to depend on the quality of cancellous bone [11]. Reportedly, patients with osteoporosis are at risk of loosening with the pedicle screws [5, 12]. The CBT screw fixation passed through vertebral pedicle from the dorsal to ventral side in the sagittal plane and from center to outside in the axial plane. The CBT screws provide maximum contact with the cortical bone, increasing the holding force between the screw and the cortical bone, which helps to add the stability of the internal screw fixation [27]. In addition, the CBT screw insertion pathway is closer to the spinous process, which enables less invasion by reducing paraspinal muscle dissection, resulting in reducing intrinsic damage and postoperative pain. In our present research, there was no CBT screw internal fixation loosening during follow-up, while one case of PS screw fixation was loosened and the bone graft fused completely after revision surgery. Meanwhile, there was a significant difference between the two groups in VAS scores for incision pain on the 1st day and 3rd day after surgery, which means that CBT realizes the minimally invasive concept.

However, there were no differences in the operative time, intraoperative blood loss, JOA score, bone grafting fusion, and complications between the CBT and PS groups. At the final follow-up, the JOA score was significantly improved in both groups compared to the preoperation. These results confirmed that both the affected-vertebra CBT screw fixation and PS fixation for lumbar TB could achieve satisfactory outcomes.

The affected-vertebra fixation through posterior CBT screw fixation combined with anterior debridement and bone grafting is a safe and effective method for lumbar TB. However, the current study has several limitations: (1) first, CBT screws have limited ability to correct kyphosis deformity and cannot be used in patients with severe kyphosis deformity (>60°); (2) second, the reliable information from all patients were difficult to obtain due to this retrospective study. Therefore, a prospective study with a larger number of patients would help confirm the advantages of the affected-vertebra fixation of CBT screw for the treatment of lumbar TB; (3) finally, the surgery is done by a central surgical team so that the results could be biased. In the future, multicenter studies with long-term follow-up data would help draw a reliable conclusion.

## 5. Conclusions

In summary, this retrospective study confirmed that both the affected-vertebra CBT screw fixation and PS fixation for lumbar TB via posterior and anterior approaches could achieve satisfactory outcomes.

## Figures and Tables

**Figure 1:** Curves of the mean visual analog scale (VAS) scores for incision pain in the groups (a) and VAS for leg pain in the groups (b). Scores range from 0 to 10, with higher scores indicating more intense pain. VAS showed a significant difference between the two groups in VAS scores for incision pain at the 1st day and 3rd day after surgery. The data are shown as the average ± SD. ^∗^*p* < 0.05.

**Figure 2:** A 54-year-old woman had lumbar 2-3 bone destruction. Her preoperative anteroposterior radiograph and CT show (a–d) that the bone destruction involved three columns. This case was treated with affected-vertebra fixation through the combined approaches including posterior CBT screw fixation and anterior debridement and bone grafting (e, f). Follow-up anteroposterior radiograph after 41 months shows good bone union (g–i). The clinical outcome was excellent.

**Figure 3:** A 64-year-old woman had lumbar 4-5 bone destruction. Her preoperative anteroposterior radiograph and CT show (a–d) that the bone destruction involved three columns. This case was treated with affected-vertebra fixation through the combined approaches including posterior PS screw fixation and anterior debridement and bone grafting (e, f). Follow-up anteroposterior radiograph after 37 months shows good bone union (g–i). The clinical outcome was excellent.

**Table 1:** Patient baseline data.

	CBT group (*n* = 27)	PS group (*n* = 25)	95% CI	*p* values
Gender (M/F)	15/12	14/11	0.984 (0.747 to 1.295)	0.974
Age (mean)	51.8 ± 9.9	52.6 ± 9.7	1.005 (0.938 to 1.076)	0.752
Number of affected segments				0.923
Single segment	14	13		
Double segments	10	10		
Triple segments	3	2		

CBT: cortical bone trajectory; PS: pedicle screw; M: male; F: female.

**Table 2:** Comparison between groups in terms of operation time, intraoperative blood loss, bone fusion time, and follow-up.

	CBT group	PS group	95% CI	*p* values
Operation time (min)	222.0 ± 12.1	229.0 ± 13.7	1.055 (0.998 to 1.114)	0.056
Intraoperative blood loss (ml)	289.7 ± 51.2	303.2 ± 34.7	1.010 (0.995 to 1.025)	0.294
Bone fusion time (mo)	3.9 ± 0.8	4.3 ± 0.9	2.084 (0.911 to 4.769)	0.104
Follow-up (mo)	40.2 ± 5.8	41.4 ± 4.2	1.067 (0.909 to 1.253)	0.394

CBT: cortical bone trajectory; PS: pedicle screw; min: minute; mo: month.

**Table 3:** Comparison of preoperation and final follow-up JOA scores for the CBT group and PS group.

	CBT group	PS group	95% CI	*p* values
Preoperation	10.6 ± 1.9	10.7 ± 2.3	0.933 (0.641 to 1.358)	0.830
Final follow-up	25.9 ± 0.9	25.4 ± 1.2	0.646 (0.338 to 1.233)	0.098
*p* values	0.000	0.000		

CBT: cortical bone trajectory; PS: pedicle screw.

## Data Availability

The datasets used or analyzed during the current study are available from the corresponding author on reasonable request.

## Abbreviations

CBT: Cortical bone trajectory
TB: Spinal tuberculosis
VAS: Visual analog scale
JOA: Japanese Orthopedic Association
PS: Pedicle screw
ESR: Erythrocyte sedimentation rate
CRP: C-reactive protein.
